The article "Intralesional Steroid Injection Versus Extracorporeal Shockwave Therapy in the Treatment of Plantar Fasciitis: A Comparative, Prospective, Case Series Study" was published in 2023. Journal: Cureus.

# Intralesional Steroid Injection Versus Extracorporeal Shockwave Therapy in the Treatment of Plantar Fasciitis: A Comparative, Prospective, Case Series Study

**DOI:** 10.7759/cureus.33593

**Published:** 2023-01-10

**Authors:** Sanjay Rai, Surbhi Rajauria, Nitish Khandelwal, Deepak C Reddy, Tej P Gupta

**Affiliations:** 1 Orthopaedics, Military Hospital Ambala, Ambala, IND; 2 Pathology and Laboratory Medicine, Maharishi Markandeshwar Institute of Medical Sciences and Research, Ambala, IND; 3 Pathology, Military Hospital Ambala, Ambala, IND; 4 Radiology, Military Hospital Ambala, Ambala, IND; 5 Orthopaedics, Base Hospital Delhi Cantt, Delhi, IND

**Keywords:** extracorporeal shockwave therapy, plantar fasciitis, ultrasound, local steroid injection, heel pain in soldiers

## Abstract

Background

This study aimed to compare and evaluate the outcomes of intralesional steroid injections (ultrasound-guided) versus extracorporeal shockwave therapy in the treatment of plantar fasciitis.

Methodology

Between January 2021 and March 2022, 120 (84 male, 36 female) patients with a confirmed diagnosis of plantar fasciitis were identified. Subjective assessment was done using Mayo Clinical Score, and objective evaluation was done by measuring plantar fascia thickness using ultrasonography. For this study, two groups were made, wherein group A was administered a high dose of extracorporeal shockwave therapy, and group B was administered ultrasound-guided intralesional or local steroid injections.

Results

Plantar fascia thickness was considerably reduced after therapy in both groups; however, the difference in thickness reduction was not statistically significant between both groups. Mayo Clinic Scores showed statistically significant improvement in pain; however, the difference in pain reduction was not statistically significant between both groups.

Conclusions

A considerable clinical and radiological improvement was noted in both groups; however, we did not record statistically significant and superior results in either group. Intralesional steroid injections provided faster clinical improvement and better patient compliance.

## Introduction

The majority of chronic heel pain is usually caused by plantar fasciitis [1]. Plantar fasciitis is a degenerative condition of the plantar fascia that affects up to 10% of the general population and about 2.5 million people per year in the United States [2]. However, data from India is not clear, especially among soldiers. Riddle and Schappert estimated that plantar fasciitis accounts for 11-15% of all foot complaints [3]. Scher et al. recorded the overall unadjusted incidence rate of plantar fasciitis as 10.5 per 1,000 person-years in the US Military [4]. This condition is associated with significant morbidity in the form of pain while standing or walking.

The article "Intralesional Steroid Injection Versus Extracorporeal Shockwave Therapy in the Treatment of Plantar Fasciitis: A Comparative, Prospective, Case Series Study" was published in 2023. Journal: Cureus.

Plantar fasciitis is caused by degenerative irritation and microscopic tearing of the plantar fascia and its surrounding perifascial structures. The plantar fascia pulling away from its insertion results in a painful heel. Repeated microtrauma and continuous pulling cause new bone formation which appears as calcaneum spur on the X-ray. It is a common belief that the calcaneum/heel spurs cause heel pain, while it is caused by the inflammation or irritation of the plantar fascia [5].

Plantar fasciitis is characterized by heel pain at the calcaneum origin of the plantar fascia, which is usually severe while getting up in the morning or after a long period of rest and continues during walking. The etiology is the deterioration of collagen fibers, shortening caused by changes in the collagen matrix of the plantar fascia, increased protein secretion, fibroblast proliferation, and neovascularization. Plantar fibromatosis is the main basis of this disease [6-8]. The diagnosis of plantar fasciitis is usually made by clinical examination.

Shockwave therapy has been used for many years as an alternative treatment for musculoskeletal disorders, especially for heel pain [9,10]. The treatment consists of mechanical acoustic waves that are transmitted through liquid and gaseous media. The biological and therapeutic effect is derived from the mechanical action of ultrasonic vibrations on tissues [11-14].

Shockwaves can be of two types, namely, radial and focal. Radial shockwaves are pneumatic waves that are produced by air compressors. These waves transmit radially, with lower penetrating capability into the tissue up to 3 cm, less impact (0.02-0.06 MJ/mm^2^), and limited biological effect [15]. Tadial shockwaves have been used for treating musculoskeletal disorders that are more superficial, such as tennis elbow, golfer’s elbow, and tendinopathy, with similar clinical outcomes as focal shockwaves [16]. Radial shockwaves are less effective and less intense compared to focal shockwaves. These shockwaves are known to cause the disintegration of fibrosis and calcifications and increase blood circulation in the affected area resulting in pain relief. In the present study, we used radial shockwaves.

On the contrary, focal shockwaves have high tissue penetration power of up to 10 cm and impact force (0.08-0.28 MJ/mm^2^) compared to radial shockwaves. They produce mechanical and biological effects of greater intensity, such as fibrinolysis, and induce neovascularization in tissues, thus initiating healing and reducing inflammation and pain [2-5].

The article "Intralesional Steroid Injection Versus Extracorporeal Shockwave Therapy in the Treatment of Plantar Fasciitis: A Comparative, Prospective, Case Series Study" was published in 2023. Journal: Cureus.

Several studies have been published on the effects of either local steroid injection therapy or shockwave therapy versus laser therapy in plantar fasciitis treatment [17-21]. However, the comparison between the therapeutic effects of intralesional or local steroid injection therapy versus extracorporeal shockwave therapy (ESWT) in plantar fasciitis treatment has not been studied extensively in the literature, especially among the military soldier population.

This study aimed to evaluate and compare the therapeutic effectiveness of ultrasound (USG)-guided intralesional steroid injection versus ESWT in the management of plantar fasciitis in the military soldier population.

## Materials and methods

Between January 2021 and March 2022, 120 patients (84 males, 36 females) between the age group of 19 and 45 years, otherwise healthy soldiers without any medical comorbidities, with the diagnosis of unilateral plantar fasciitis who attended the orthopaedic outpatient department were included in this study. Institutional Ethical Committee approval was obtained from Military Hospital Ambala (approval number: MHA/EC/Ortho/01/2021). The diagnosis of plantar fasciitis was made based on tenderness at the origin of the plantar fascia on the medial aspect of the heel and the presence of sharp shooting foot pain, which was worse in the morning or with activity. A full rheumatological workup including erythrocyte sedimentation rate (ESR), C-reactive protein (CRP), rheumatoid arthritis (RA) factor, human leucocyte antigen (HLA) B27, anti-cyclic citrullinated peptide (anti-CCP), and serum uric acid was done to rule out any existing inflammatory joint disease or any autoimmune arthritis like systemic lupus erythematosus, RA ankylosing spondylosis, psoriasis, gout, and inflammatory bowel disease which can cause plantar fasciitis or heel pain.

Inclusion criteria

Informed written consent was obtained from all soldiers who participated in the study. The inclusion criteria were age between 19 and 45 years, diagnosis of plantar fasciitis, and symptomatic painful heel for more than three months.

Study design

Functional assessments such as gait, footwear, and pain Mayo Clinical Score were used. The scoring system consisted of 100 points with six parameters (degree of pain, activity limitations, footwear or orthotic requirement, plantar heel tenderness, neuropathy, and antalgic gait) [16]. The results were classified as excellent with 90-100 points, good with 80-89 points, fair with 70-79 points, and poor with <70 points.

Radiological evaluation

A plain lateral view X-ray of the heel was obtained to diagnose a calcaneal spur or any pre-existing calcaneal abnormality.

The article "Intralesional Steroid Injection Versus Extracorporeal Shockwave Therapy in the Treatment of Plantar Fasciitis: A Comparative, Prospective, Case Series Study" was published in 2023. Journal: Cureus.

Ultrasound scanning and evaluation

A high-resolution USG scan was used to measure the thickness of the plantar fascia in the involved foot and on the contralateral normal foot. The thickness of the plantar fascia was measured at its thickest portion. Patients were divided into two treatment groups using the simple randomization method. Group A was administered medium-energy density (0.28 mJ/mm^2^) shockwave therapy at maximal tenderness point at two-week intervals. Group B was administered USG-guided intralesional injection in two sessions at two-week intervals.

Shockwave therapy procedure

The patient was placed in a prone position, and the foot was fixed with a foot holder. Shockwaves were administered using an electrohydraulic shockwave machine (EWST machine, Class I Type BF, Electronica PAGANI, Italy). The probe of the shockwave device was placed on the most painful point of the proximal heel, and two series of shocks were applied. The energy between 14 and 17 kV, 2 Hz, and 1,000-1,500 pulses were applied in two directions to cover the maximum painful area. Two sessions were given once per week for two weeks (Figure 1).

**Figure 1:** Extracorporeal shockwave therapy being delivered to a patient.

Intralesional injection procedure

Intralesional injections for group B were administered under aseptic conditions. In a prone position at the most tender point, the needle was inserted through the medial aspect of the heel using a USG transducer. The needle was advanced until it reached the plantar fascia, and then the drug was injected. Two injections of 1 mL 40 mg/mL (methylprednisolone acetate) combined with an intralesional anesthetic agent (1 mL of 2% xylocaine hydrochloride) were administered and repeated after two weeks. Care was taken to avoid injecting into the fat pad.

Evaluation

We recorded the data before the treatment, immediately after the procedure, and three months after treatment. We recorded (a) pain assessment using the Visual Analog Scale (VAS) for morning pain, painful gait pain, and orthostatic pain; (b) use of non-steroidal anti-inflammatory drugs (NSAIDs) during treatment; (c) periodicity of heel pain (the number of times each week that patients experienced pain); and (d) duration of pain (the number of hours each day in a week) by an independent observer. The follow-up period was three months.

Statistical analysis

The data were collected and tabulated. We used SPSS software version 19 (IBM Corp., Armonk, NY, USA) for statistical analysis. Paired-sample Student’s t-test was performed to compare two numerical variables (before and after treatment). To compare two groups regarding numerical variables an independent-sample Student’s t-test was performed. We used the Pearson correlation coefficient to assess the linear association between two numerical variables.

The article "Intralesional Steroid Injection Versus Extracorporeal Shockwave Therapy in the Treatment of Plantar Fasciitis: A Comparative, Prospective, Case Series Study" was published in 2023. Journal: Cureus.

## Results

The demographic characteristics of the patients are shown in Table 1. We did not record any significant differences in demographic characteristics such as age, sex, or body mass index.

**Table 1:** Demographic data of the two treatment groups. ESWT = extracorporeal shockwave therapy; USG = ultrasound; M/F = male/female; BMI = body mass index; t = Student’s t-test

Characteristics	Group A (ESWT), N = 60	Group B (USG-guided onsite injection), N = 60	T	P-value
Mean age (years)	40.43 ± 4.154	41.42 ± 4.238	-0.018	0.975
Sex (M/F)	43/27	38/22		
BMI (kg/m²)	27.801 ± 2.512	28.236 ± 2.845	-0.607	0.536
Height (in cm)	172 ± 32. 31	169 ± 52.18	-0.512	0.742
Smoking	17	23	-	0.763
Alcoholism	11	9	-	0.667

Occupation of both groups and standing time per day did not show any significant differences; however, the majority of individuals had more than six hours of standing duty per day, as shown in Table 2.

**Table 2:** Occupation of study groups and standing time per day.

Occupation	Group A, N = 60	Group B, N = 60	Standing time at a stretch in 24 hours
Security guard	18	12	More than 6 hours
Repeated parading and constant walking	7	10	More than 6 hours
Watchtower duty	14	19	More than 7 hours
Office job	9	7	Fewer than 5 hours
Sedentary job/household work	12	12	Fewer than 3 hours

Subjective assessment was done using the Mayo Clinic Scoring system at the end of 12 weeks of follow-up, and objective evaluation was done by measuring the thickness of the plantar fascia. The data obtained were analyzed. In group A (ESWT group), a significant reduction in the thickness of the plantar fascia was noted from 4.566 ± 0.436 before treatment to a mean of 3.5783 ± 0.31 after treatment (t = -38.36, p < 0.001) (Table 3).

**Table 3:** Comparison between planter fascia thickness and Mayo CSS pre- and post-treatment in group A at three months. Mayo CSS = Mayo Clinical Scoring System; t = Student’s t-test

Parameters	Before treatment	After treatment	t	P-value
Planter fascia thickness	4.566 ± 0.436	3.5783 ± 0.31	-38.36	<0.001
Mayo CSS	46.66 ± 10.44	74.00 ± 6.61	-23.549	<0.001

In group B (onsite injection group), a significant reduction in the thickness of plantar fascia was noted from a mean of 5.78 ± 0.556 before treatment to a mean of 3.45 ± 0.41 after treatment (t = -22.469, p < 0.00) (Table 4).

**Table 4:** Comparison between planter fascia thickness and Mayo CSS pre- and post-treatment in group B at three months. Mayo CSS = Mayo Clinical Scoring System; t = Student’s t-test

Parameters	Before treatment	After treatment	T	P-value
Planter fascia thickness	5.78 ± 0.556	3.45 ± 0.41	-22.469	<0.001
Mayo CSS	43.67 ± 10.48	82.23 ± 7.63	-24.413	<0.001

The number of pain hours per day before and after treatment in both groups is shown in Table 5.

The article "Intralesional Steroid Injection Versus Extracorporeal Shockwave Therapy in the Treatment of Plantar Fasciitis: A Comparative, Prospective, Case Series Study" was published in 2023. Journal: Cureus.

**Table 5:** Number of hours of pain per day in groups A and B before and after treatment. Friedman test – intragroup evaluation. Analysis of variance – intergroup evaluation. ESWT = extracorporeal shock wave therapy; USG = ultrasound

Number of hours of heel pain per day	Group A (ESWT), N = 60			Group B (USG-guided local injection), N = 60		
	Pretreatment	At 0 months	At 3 months	Pretreatment	At 0 months	At 3 months
0 hours	0 (0%)	19 (31.6%)	24 (40%)	0 (0%)	22	34
>4 hours	27 (45%)	29 (48.3%)	33(55%)	24	36	15
Up to 4 hours	33 (55%)	12(20%)	2(3%)	36	2	1
P-value*		0.001			0.002	

Data regarding the intensity of antalgic gait as per VAS in both groups before and after treatment is shown in Table 6.

**Table 6:** Patient data regarding intensity of antalgic gait as per the VAS in both groups before and after treatment. Friedman test – intragroup evaluation. Analysis of variance – intergroup evaluation. ESWT = extracorporeal shock wave therapy; USG = ultrasound; VAS = Visual Analog Scale

VAS	Group A (ESWT), N = 60			Group B (USG-guided onsite injection), N = 60		
	Pretreatment	At 0 day	At 3 months	Pretreatment	At 0 day	At 3 months
Good (0–1)	1 (1.6%)	19 (31.6%)	18 (30%)	1 (1.6%)	22 (36.6)	39 (62.9)
Regular (2–5)	18 (30%)	33 (55%)	38 (66.3%)	11 (18.3%)	36 (60%)	20 (33.3%)
Poor (6–10)	41 (68.3%)	8 (13.3%)	4 (6.6%)	48 (80%)	2 (3.3%)	1 (1.6%)
P-value*		<0.001	<0.001		<0.002	<0.001

Data regarding orthostatic pain as per VAS in both groups before and after treatment is shown in Table 7.

**Table 7:** Patient data regarding the intensity of orthostatic pain as per VAS in both groups before and after treatment. Friedman test – intragroup evaluation. Analysis of variance – intergroup evaluation. ESWT = extracorporeal shock wave therapy; USG = ultrasound; VAS = Visual Analog Scale

VAS	Group A (ESWT), N = 60			Group B (USG-guided onsite injection), N = 60		
	Pretreatment	At 0 day	At 3 months	Pretreatment	At 0 day	At 3 months
Good (0–1)	-	16 (26.6%)	41 (68.3%)	-	19 (22.6%)	40 (66.6%)
Regular (2–5)	3 (5%)	26 (43.3%)	17 (28.3%)	7 (11.6%)	23 (38.8%)	15 (25%)
Poor (6–10)	57 (95%)	18 (30%)	2 (3.3%)	43 (71.4%)	18 (30%)	5 (8.3%)
P-value*		<0.001	<0.001		<0.002	<0.001

Data regarding the intensity of morning pain as per VAS in both groups before and after treatment is shown in Table 8.

**Table 8:** Patient data regarding the intensity of morning pain as per VAS in both groups before and after treatment. Friedman test – intragroup evaluation. Analysis of variance – intergroup evaluation. ESWT = extracorporeal shock wave therapy; USG = ultrasound; VAS = Visual Analog Scale

VAS	Group A (ESWT), N = 60			Group B (USG-guided onsite injection), N = 60		
	Pretreatment	At 0	At 3	Pretreatment	At 0	At 3
Good (0–1)	0 (0%)	9 (15%)	27 (45%)	2 (3.3%)	29 (48.3%)	44 (73.3)
Regular (2–5)	11 (18.3%)	35 (58.3%)	24 (40%)	17 (28.3%)	26 (43.3%)	14 (23.3%)
Poor (6–10)	49 (81.6%)	16 (26.6%)	9 (15%)	41 (66.6%)	5 (8.3%)	2 (3.3%)
P-value*		0.002	<0.001		<0.001	<0.001

Data regarding the periodicity of heel pain as per VAS before and after treatment did not show any significant difference between both treatment groups (Table 9).

The article "Intralesional Steroid Injection Versus Extracorporeal Shockwave Therapy in the Treatment of Plantar Fasciitis: A Comparative, Prospective, Case Series Study" was published in 2023. Journal: Cureus.

**Table 9:** Patient data regarding the periodicity of heel pain as per VAS in both groups before and after treatment. ESWT = extracorporeal shock wave therapy; USG = ultrasound; VAS = Visual Analog Scale

VAS score	Periodicity of pain	Group A (ESWT)			Group B (USG-guided onsite injection)		
		Pretreatment	At 0 day	At 3 months	Pretreatment	At 0 day	At 3 months
6–10	Morning pain only	60	36	4*	60	29	2*
2–5	Mid-day pain	42	15	11	33	23	11
1–0	Evening pain	26	9	19	43	18	15
1–0	Throughout the day	68	24	30	76	41	26
*P-value				<0.001			<0.001

Subjective analysis was done according to the Mayo Clinic Scoring System. Patients in the ESWT group (group A) showed a significant improvement from 46.66 ± 10.44 before ESWT to a mean of 74.00 ± 6.61 after ESWT (t = -23.549, p < 0.001), with 49 (81%) patients having excellent scores. Similarly, the USG-guided injection group (group B) also showed statistically significant improvement from a mean of 43.67 ± 10.48 before injection to a mean of 82.23 ± 7.63 after injection (t = -24.413, p < 0.001), with 54 (90%) patients having excellent scores, as shown in Table 10.

**Table 10:** Comparison of Mayo CSS in both group pre- and post-treatment at three months. Mayo CSS = Mayo Clinical Scoring System; t = Student’s t-test

Parameters	Group	Before treatment	After treatment	t	P-value
Mayo CSS	A (n = 49/60) 81%	46.66 ± 10.44	74.00 ± 6.61	-23.549	<0.001
Mayo CSS	B (n =54/60) 90%	43.67 ± 10.48	82.23 ± 7.63	-24.413	<0.001

We did not find any significant difference in the plantar fascia thickness in groups A and B before and after treatment (t = 0.154, p = 0.879, and t = 1.79, p = 0.078, respectively). Similarly, the Mayo Clinical Scoring System scores between the two treatment groups before and after treatment failed to show any significant differences (t = -0.064, p = 0.949 and t = -1.056, p = 0.296, respectively).

The Pearson correlation analysis showed a significant positive association between the plantar fascia thickness before treatment and BMI (rA = 0.410, PA < 0.05, and rB = 0.389, PB < 0.05, respectively), and a significant negative correlation between plantar fascia thickness before treatment and the Mayo scores before treatment (rA = 0.6812 rB = 0681, respectively, and PA = 0.001, PB = 0.001, respectively).

The article "Intralesional Steroid Injection Versus Extracorporeal Shockwave Therapy in the Treatment of Plantar Fasciitis: A Comparative, Prospective, Case Series Study" was published in 2023. Journal: Cureus.

At a mean follow-up of five months (range = 3-6 months), 93% of patients in both treatment groups showed good to excellent results according to the Mayo Clinic Scoring System. Three patients in group A and five patients in group B (n = 8, 6%) showed poor or unsatisfactorily responses to treatment and were subsequently managed by surgical release of the plantar fascia. Seven patients from group A and 11 patients from group B (n = 18, 15%) showed recurrence of symptoms of plantar fasciitis within two months after the last treatment. The time before recurrence ranged from two months to six months (mean of four months).

## Discussion

The medial longitudinal arch of the foot is supported by the plantar fascia, and it becomes inflamed due to repetitive microtrauma at its origin of the medial tuberosity of the calcaneus. Generally, traction forces during support lead to inflammation, which, in turn, leads to fibrosis and degeneration [22]. Allam and Chang reported that calcaneal/heel spurs and nerve trappings (medial calcaneal, lateral plantar) can be associated with the inflammatory process [23].

Although both men and women are affected equally, sometimes women are more often affected than men. Plantar fasciitis is sometimes associated with obesity and the climacteric [24]. In this study, men were more frequently affected than women (81% vs. 19%) because they were mostly working outdoors and doing more prolonged standing work. Those who were slightly overweight (4.2%) were also more affected.

Plantar fasciitis seems to be related to the occupation of the individual and activities such as sports, standing for a longer time, parades, drills, repeated jumps, and long rout marchpast, which require constant support of body weight. Most soldiers in this study (66.6%) performed their work while standing (security guard, marchpast, and watch guards), and stood for more than six hours a day every day. It indicates the mechanical factors that play a crucial role in the etiopathogenesis of this disease. We did not record any loss of strength in the Achilles tendon or ankle planter and dorsiflexion post-treatment.

Pribut [25] reported that steroid injection and ESWT were successful treatment modalities for plantar fasciitis. He also noted that local corticosteroid injection treatment was cost-effective compared with ESWT, with steroid injection being the first treatment choice. In our study, morning pain was reported by 81% of the patients, antalgic gait by 64%, and orthostatic pain by 82%. These findings are similar to those of other published studies [17,26,27-29]. The presence of morning pain is an important evaluation criterion in management. In our study, regarding the intensity of morning pain, the mean VAS score was 7 (range = 4-10) and 3 (range = 1-5) in pre-treatment and post-treatment, respectively. After treatment, 109 out of 120 (90%) patients in both groups had VAS scores of less than 5, indicating that both treatments were equally effective in alleviating pain at the end of the three-month follow-up.

The article "Intralesional Steroid Injection Versus Extracorporeal Shockwave Therapy in the Treatment of Plantar Fasciitis: A Comparative, Prospective, Case Series Study" was published in 2023. Journal: Cureus.

In this study, we noted a statistically significant reduction in plantar fascia thickness after treatment at 12 weeks, as measured by USG in both groups. This reduction in plantar fascia thickness was more in the ESWT group compared to the local injection group. Regarding the reduction of heel pain, our results are supported by Porter and Shadbolt [30] and Tsai et al. [31], who reported that ESWT and steroid injection showed significant improvements in VAS and heel tenderness index scores; however, after three months of treatment, there was no significant difference in the VAS score.

A study by Yucel et al. [32] compared high-dose ESWT and intralesional steroid injection in the treatment of plantar fasciitis. Two groups were treated and showed significant improvements in VAS and heel tenderness index scores; however, there was no significant difference after three months of treatment. Saber et al. [33] divided 60 patients into two equal groups, with one group receiving local steroid injections (two doses two weeks apart) and the other group receiving shockwave therapy (two sessions and two weeks apart). In their study, both groups showed good clinical and radiological improvement in plantar fasciitis. Further, they recommended local steroid injections for faster pain relief.

On the other hand, some studies have reported conflicting results. Grice et al. [34] reported that local steroid injections showed a lesser effect on pain relief at 12 weeks after injection. On the contrary, McMillan et al. [35] reported that local steroid injection exhibited greater pain relief at four weeks and a significant reduction in the plantar fascia thickness at three months compared with the placebo group.

More recently, Xu et al. [36] in a randomized controlled study compared 49 patients treated with ESWT and 47 patients treated with local steroid injection and recorded that both ESWT and local steroid injection had similar clinical improvement; however, EWST provided longer pain relief than local steroid injection. Polat et al. [37] in 56 patients noted that ESWT and local corticosteroid injection are effective in pain relief in patients with chronic plantar fasciitis with a calcaneal spur. Further, they concluded that local steroid injections seem to be more effective for pain relief compared to ESWT.

The article "Intralesional Steroid Injection Versus Extracorporeal Shockwave Therapy in the Treatment of Plantar Fasciitis: A Comparative, Prospective, Case Series Study" was published in 2023. Journal: Cureus.

Ogden et al. [38] noted several issues with ESWT such as shockwave dosage, high- versus low-energy ESWT, and the number of sessions required for pain relief. However, some studies have ascertained that the efficacy of ESWT may be highly dependent upon the type of machine and treatment protocols [39,40]. After a review of the literature, we can conclude that more investigation needs to be done to determine the optimal and appropriate protocols, especially in the military soldier population, for the use of shockwave therapy in plantar fasciitis.

Study limitations

This study was done among soldiers who did not have any comorbidities, and the results obtained may not be applicable to the general population. We are not sure whether similar results can be obtained with patients with other medical comorbidities. A larger study is required on this subset of people (soldiers) to formulate guidelines and the effectiveness of these treatments.

## Conclusions

We can conclude that both ESWT and the intralesional or local steroid injections are equally effective in the management of plantar fasciitis. Both modes of therapy showed significant clinical improvement, and USG documented improvement after therapy with slightly superior results in the ESWT group. Intralesional steroid injection is a preferred method being more economical and more patient compliance. However, ESWT should be considered before any invasive therapy such as the surgical release of the plantar fascia or any other intervention for non-responsive plantar fasciitis.
